# Clinical significance of SPOCK2 expression signature for high-grade serous ovarian cancer patients

**DOI:** 10.3389/fgene.2022.878123

**Published:** 2022-09-28

**Authors:** Mi Jiao, Wenbo Sun, Lina Li, Chunyan Li, Jing Zhou, Qian Li, Lian Duan

**Affiliations:** ^1^ Xi’an Jiaotong University Health Science Center, Xi’an Jiaotong University, Xi’an, Shaanxi, China; ^2^ Department of Medical Oncology, Shaanxi Provincial Cancer Hospital Affiliated to Xi’an Jiaotong University Medical College, Xi’an, Shaanxi, China

**Keywords:** SPOCK2, high-grade serous ovarian cancer (HGSOC), biomarker, prognosis, extracellular matrix, tumor infiltrating lymphocytes (TILs)

## Abstract

**Background:** SPOCK2 is a member of the SPOCK family, a 424-amino acid protein that binds to glycosaminoglycans to form proteoglycans. The purpose of this study was to explore expression profile of SPOCK2, and evaluate prognostic potential and its correlation with immune infiltration in high-grade serous ovarian cancer (HGSOC).

**Methods:** Expression of SPOCK2 mRNA and protein between normal and tumor tissues were analyzed using the Cancer Genome Atlas database (TCGA), Gene Expression Omnibus (GEO), Clinical Proteomic Tumor Analysis Consortium (CPTAC), and the Human Protein Atlas (HPA) databases. Receiver operating characteristic (ROC) curve was used to evaluate diagnostic performance of SPOCK2. Kaplan-Meier method and Cox regression analysis were conducted to assess the effect of SPOCK2 on survival. Nomogram was used to predict the impact of SPOCK2 on prognosis. LinkedOmics were used to find correlated genes and perform functional enrichment analyses. The relationships between SPOCK2 and tumor infiltrating lymphocytes (TILs) were determined by tumor-immune system interaction database (TISIDB) and GSVA package (V1.34.0).

**Results:** SPOCK2 was highly expressed in HGSOC tissue compared to normal tissue at both mRNA (*p* < 0.001) and protein (*p* = 0.03) levels. The area under the curve (AUC) is 0.894 (CI: 0.865–0.923). Kaplan-Meier analysis showed that HGSOC patients with high-level SPOCK2 mRNA expression had a worse overall survival (OS) than those with a low expression (HR = 1.45, *p* = 0.005). Univariate logistic regression analysis found that age, primary therapy outcome, tumor status, tumor residual, and SPOCK2 expression level were significantly associated with OS (*p* < 0.05). The nomogram model indicated an effective predictive performance of SPOCK2. Kyoto encyclopedia of genes and genomes (KEGG) and gene ontology (GO) term analyses showed that SPOCK2 were mainly involved in regulating extracellular matrix. Immune infiltration analysis showed that SPOCK2 may correlate with abundance of TILs.

**Conclusion:** SPOCK2 has potentials to estimate diagnosis and prognosis for HGSOC and is involved in regulating extracellular matrix and immune cell infiltration.

## Introduction

High-grade serous ovarian cancer (HGSOC) is of particular interest, as it comprises over 70% of epithelial ovarian cancer (EOC) and accounts for the majority of deaths within the first 3 months of ovarian cancer diagnoses, indicating high morbidity and mortality that caused by late-stage presentation and insufficient therapies (Lheureux et al., 2019; Kuroki and Guntupalli, 2020). About 75% of newly-diagnosed EOC patients are at an advanced stage due to a lack of early and typical warning signs or symptoms as well as effective screening strategies, with 20%–40% 5-years survival (Reid et al., 2017; Kurnit et al., 2021; Huang et al., 2022). Although debulking surgery and platinum/taxane-based chemotherapy regimens are given to delay disease progression or cure the cancer, approximately 70% of all ovarian cancer patients will succumb to the disease to enter a recurrent or relapse setting (Einzig et al., 1992; Hamanishi et al., 2015; Lheureux et al., 2019). In addition to systemic therapy that maximizes the effect of killing cancer cells in a platinum-sensitive setting, poly (ADP-ribose) polymerase inhibitors (PARPi) have presented remarkable benefit in women with recurrent HGSOC regardless of BRCA mutation status, by contrast with improved activity in patients harboring BRCA mutations and platinum-sensitive disease (Mirza et al., 2016; Oza et al., 2018; González-Martín et al., 2019). Nevertheless, multiple acquired resistance mechanisms to PARPi and potential drug toxicities have retarded clinical efficacy, suggesting that efforts might be leveraged into novel researches to delineate resistance mechanisms, prompt drug responses, or find new and specific prognostic biomarkers and therapeutic targets (Kubalanza and Konecny 2020; Hao et al., 2021).

SPARC (osteonectin), cwcv and kazal-like domains proteoglycan 2 (SPOCK2), also known as testican-2, is a member of the SPARC family composing of FSTL1, SMOC1, SMOC2, SPARC, SPARCL1, SPOCK1, SPOCK2, and SPOCK3 (Said et al., 2008; Bradshaw, 2012). The protein encoded by SPOCK2 gene contains thyroglobulin type 1, follistatin-like, and calcium-binding domains as well as glycosaminoglycan binding sites in the acidic C-terminal region, which contribute to form a glycoprotein to orchestrate extracellular matrix and cell membranes (Vannahme et al., 1999). In addition to modulating extracellular matrix formation, SPOCK2 can serve as receptors for growth factors and regulate cellular differentiation and growth (Vannahme et al., 1999). Furthermore, abnormal expression of SPOCK2 have been correlated with tumor growth, invasion, and migration in various human cancers. Previous studies reported that upregulation of SPOCK2 can decrease invasion and metastasis of prostate cancer and endometrial cancer by inhibiting matrix metalloproteinase 2 (MMP2) and membrane-type 1 matrix metalloproteinase (MT1-MMP) (Liu et al., 2019; Ren et al., 2020). Efforts have been made to understand the role of SPOCK2 in tumorigenesis, yet the relationship between SPOCK2 and anti-tumor immunity should also be investigated because extracellular matrix was reported to regulate immune microenvironment surrounding the tumor mass (Sorokin, 2010; Crespo et al., 2018). Therefore, studies must be conducted to address the functional contribution of SPOCK2 to tumor immunity, particularly in ovarian cancer.

To incorporate extracellular matrix on cancer immunity and prognosis in HGSOC, we could proceed with SPOCK2. In this study, we first evaluated the patient characteristics and expression of SPOCK2 using the Cancer Genome Atlas (TCGA) and Genotype Tissue Expression (GTEx) datasets, and subsequently examined association between clinical features and prognostic significance of SPOCK2 using Cox regression analysis. Furthermore, we explored the positively and negatively correlated genes of SPOCK2 in HGSOC, and conducted kyoto encyclopedia of genes and genomes (KEGG) pathway analysis and gene ontology (GO) term analysis. Finally, the impact of SPOCK2 on tumor infiltrating immune cells were analyzed. Our study is important in improving understandings of SPOCK2 in HGSOC and finds that SPOCK2 might be a potential prognostic and therapeutic biomarker for HGSOC.

## Material and methods

### Data acquisition and preprocessing

RNA-seq transcriptomic data of normal and tumor tissues were respectively downloaded from GTEx and TCGA datasets using UCSC XENA (https://xenabrowser.net/datapages/) to analyze expression level of SPOCK2. The RNA-seq data with workflow type of HTSeq-FPKM (high throughput sequencing-fregments per kilobase per million) were transformed to TPM (transcription per million reads) format which was processed *via* the Toil procedure (Vivian et al., 2017), and the subsequent log2 conversions were performed for the following analyses. Furthermore, the corresponding patients’ clinical information from HGSOC samples were downloaded from TCGA dataset (https://portal.gdc.cancer.gov). Since all gene expression data and patient information were downloaded using R (V3.6.3), the consent from the Ethics and Committee was waived.

### Differential expression of SPOCK2

The ggplot2 package (V3.3.3) was used to visualize differential expression of SPOCK2. RNA sequencing data of 8,295 normal and 9,807 tumor tissues was preprocessed, and the Wilcoxon rank sum test was applied to analyze pan-cancer expression level of SPOCK2 in non-paired samples. The Weltch t' test was subsequently used to assess the differential mRNA expression of SPOCK2 between 88 normal ovary tissues and 427 HGSOC samples. In addition, we performed UALCAN (http://www.ualcan.path.uab.edu/analysis.html) to present differential mRNA expression of SPOCK2 according to clinical features (Chandrashekar et al., 2017). To identify protein profile of SPOCK2 between normal ovary tissues and HGSOC samples, the human protein atlas (HPA) (https://www.proteinatlas.org) was used to download immunohistochemical images. With the application of proteomic technologies, we used the clinical proteomic tumor analysis consortium (CPTAC) (http://www.ualcan.path.uab.edu/analysis-prot.html) to quantify SPOCK2 protein and find associations of SPOCK2 protein level with clinical features (Edwards et al., 2015). The association between SPOCK2 mRNA expression level and clinical characteristics were analyzed with Fisher test or Chi-square test and logistic regression. The diagnostic role of SPOCK2 in HGSOC was assessed by receiver operating characteristic (ROC) curve analysis based on TCGA data.

### Western blotting

Protein samples were prepared from the ovarian cancer cell lines. Protein concentration was determined with Bradford protein assay reagent using BSA as the standard. Protein (20 µg) was separated by 12% SDS-PAGE, transferred to a polyvinylidene fluoride (PVDF), and blocked with 5% fat-free milk in TBST at room temperature for 1 h. The membranes were incubated at 4°C overnight with the monoclonal antibody against SPOCK2 (1:1,000 dilution, Santa Cruz Biotechnology, Texas, United States) and Actin (1:10,000 dilution, Wuhan Sanying, Wuhan, China) from mouse. Membranes were then incubated with horseradish peroxidase (HRP)-conjugated anti-rabbit and anti-mouse antibodies (1:4,000 dilution, Proteintech, Wuhan, Hubei, China) at room temperature for 1 h. An enhanced chemiluminescence (NCM Biotech, Suzhou, China) detection system (Bio-Rad) was used to visualize immunoreactive bands. The densitometry of each protein band was quantified using ImageJ 1.46r software (NIH, Bethesda, MD, United States).

### Statistical analysis on prognosis of SPOCK2

The survminer package (V0.4.9) was used to evaluate prognostic potential of SPOCK2 and the cut-off point of SPOCK2 expression was determined by its median value. To investigate the effect of SPOCK2 expression level along with other clinical factors (age, race, FIGO stage, and histologic grade) on OS in TCGA patients, the Kaplan-Meier method with a two-sided log-rank test was used. Furthermore, the survival package (V3.2-10) and the Cox regression analysis was applied to calculate the effect of SPOCK2 expression level and other clinicopathological features (age, race, FIGO stage, histologic stage, primary therapy outcome, tumor status, tumor residual, lymphatic invasion, venous invasion, and anatomic neoplasm subdivision) on survival. The independent prognostic factors derived from multivariate analysis were employed to predict 1-, 3-, and 5-years survival probability, which were visualized using a nomogram. Moreover, the nomogram-predicted probabilities were graphically demonstrated by calibration curves. The concordance index (C-index) was used to assess the discrimination of the nomogram, which was calculated by a bootstrap approach with 1,000 resamples. Notably, nomograms and calibration curves were generated by the rms (V6.2-0) and survival (V3.2-10) packages. All statistical tests were considered as significant if *p*-values were less than 0.05.

### Co-expressed genes and functional enrichment

LinkedOmics (http://www.linkedomics.org/login.php) is a publicly available dataset that contains multi-omics data from all 32 cancer types and a total of 11,158 TCGA patients (Vasaikar et al., 2018). The web application has three analytical modules including LinkFinder, LinkInterpreter, and LinkCompare. Co-expressed genes related to SPOCK2 were identified from the TCGA-OV cohort through the LinkFinder module. The association results were examined by the Pearson correlation coefficient and a Z-score, which were presented in a volcano plot and heat maps, respectively. In the LinkInterpreter module, functional enrichment analyses of KEGG and GO pathways by the gene set enrichment analysis (GSEA) were performed.

### Analysis of immune cell infiltration

We first construct an overall insight of immune cell infiltration related to SPOCK2 using TISIDB (http://www.cis.hku.hk/TISIDB/index.php) which is a web portal for tumor-immune system interactions and integrates multiple heterogeneous data types (Ru et al., 2019). In this study, we performed TISIDB to determine relations between abundance of tumor infiltrating lymphocytes (TILs) and expression level of SPOCK2 across human cancers. For HGSOC, the relative abundance of 24 immune cell types based on SPOCK2 expression profile was inferred by using ssGSEA that was incorporated in the GSVA package (V1.34.0). To explore the correlation between SPOCK2 mRNA expression level and the enrichment of TILs, scatter plots and Spearman correlation were adopted. Finally, a *t* test was applied to examine the difference of enrichment score of immune cells between SPOCK2-low and -high groups. All statistical tests were two tailed with a statistical significance level cut-off at 0.05.

## Results

### Pan-cancer analyses of SPOCK2 expression

We first carried out pan-cancer analyses to evaluate the SPOCK2 mRNA expression profile in the tumor samples of TCGA and the normal samples of GTEx combined with TCGA across different cancer types. The differential expression analyses of SPOCK2 mRNA was finally referred to 33 cancer types by using Wilcoxon rank sum test (Figure 1). Compared with normal tissues, SPOCK2 was significantly upregulated in breast infiltrating carcinoma (BRCA), cholangiocarcinoma (CHOL), diffuse large B cell lymphoma (DLBCL), esophageal carcinoma (ESCA), head and neck squamous cell carcinoma (HNSC), acute myeloid leukemia (LAML), brain low grade glioma (LGG), liver hepatocellular carcinoma (LIHC), ovarian serous cystadenocarcinoma (OV), pancreatic cancer (PAAD), pheochromocytoma and paraganglioma (PCPG), skin melanoma (SKCM), gastric cancer (STAD), thyroid cancer (THCA), thymic cancer (THYM), endometrial cancer (UCEC), uterine sarcoma (UCS) (*p* < 0.05); by contrast, SPOCK2 was significantly downregulated in adrenocortical carcinoma (ACC), colon adenocarcinoma (COAD), pleomorphic glioma (GBM), renal chromophobe cell carcinoma (KICH), renal clear cell carcinoma (KIRC), renal papillary cell carcinoma (KIRP), lung adenocarcinoma (LUAD), lung squamous cell carcinoma (LUSC), rectum adenocarcinoma (READ), testicular germ cell tumors (TGCT) (*p* < 0.05).

**FIGURE 1:** Transcription level of SPOCK2 in pan-cancer perspective. ACC, adrenocortical carcinoma; BLCA, bladder urothelial carcinoma; BRCA, breast infiltrating carcinoma; CESC, cervical squamous cell carcinoma; CHOL, cholangiocarcinoma; COAD, colon adenocarcinoma; DLBCL, diffuse large B cell lymphoma; ESCA, esophageal carcinoma; GBM, pleomorphic glioma; HNSC, head and neck squamous cell carcinoma; KICH, renal chromophobe cell carcinoma; KIRC, renal clear cell carcinoma; KIRP, renal papillary cell carcinoma; LAML, acute myeloid leukemia; LGG, brain low grade glioma; LIHC, liver hepatocellular carcinoma; LUAD, lung adenocarcinoma; LUSC, lung squamous cell carcinoma; MESO, mesothelioma; OV, ovarian serous cystadenocarcinoma; PAAD, pancreatic cancer; PCPG, pheochromocytoma and paraganglioma; PRAD, prostate adenocarcinoma; READ, rectum adenocarcinoma; SARC, sarcoma; SKCM, skin melanoma; STAD, gastric cancer; TGCT, testicular germ cell tumors; THCA, thyroid cancer; THYM, thymic cancer; UCEC, endometrial cancer; UCS, uterine sarcoma; UVM, uveal melanoma. (Significant codes of *p*-value: ns, *p* ≥ 0.05; *, *p* < 0.05; **, *p* < 0.01; ***, *p* < 0.001).

### Upregulated expression of SPOCK2 in high-grade serous ovarian cancer

To analyze the mRNA and protein expression level of SPOCK2 in HGSOC, we compare the expression data from TCGA and HPA datasets. The non-paired data analysis found that the mRNA expression level of SPOCK2 in 427 TCGA HGSOC samples was significantly higher than those in 88 GTEx normal ovarian samples (5.265 ± 1.691 vs. 2.795 ± 1.008, *p* < 0.001, Figure 2A). Moreover, a CPTAC analysis was performed to verify the proteomic expression profile of SPOCK2. Compared with 25 normal tissues, 100 ovarian cancer samples were found to have a comparatively higher level of SPOCK2 protein expression (*p* = 0.03, Figure 2B). As shown in Figures 2D,E, the immunohistochemical staining images from HPA, on the other hand, confirmed that SPOCK2 protein was upregulated in ovarian cancer tissue. Furthermore, the results of western blotting indicated that ovarian cancer cell lines including A2780, CaoV-3, OVCAR3, and SKOV-3 expressed higher levels of SPOCK2 protein, compared with IOSE80 (Figure 2F). In general, these results indicated that both mRNA and protein expression levels of SPOCK2 were upregulated in HGSOC. In addition, the ROC curve was used to determine the distinguishing efficacy of SPOCK2 between normal ovarian tissues (*n* = 88) and HGSOC tissues (*n* = 427) (Figure 2C). The area under the curve (AUC) of SPOCK2 is 0.894 (CI: 0.865–0.923), suggesting that SPOCK2 is a potential identification marker for HGSOC tissues.

**FIGURE 2:** Expression profile and diagnostic performance of SPOCK2 in high-grade serous ovarian cancer (HGSOC). Expression level of SPOCK2 mRNA **(A)**. Expression level of SPOCK2 protein **(B)**. Receiver operating characteristic (ROC) curve for SPOCK2 **(C)**. Protein levels of SPOCK2 in ovary tissue and ovary carcinoma based on Human Protein Atlas (HPA) **(D–F)**. (Significant codes of *p*-value: *, *p* < 0.05; ***, *p* < 0.001).

### Relationships between SPOCK2 expression and clinical features

In order to evaluate the relationships between expression level of SPOCK2 and clinical pathological characteristics of ovarian cancer samples, we used UALCAN for differential analysis, which found that SPOCK2 was significantly associated with clinical features on transcriptional and translational levels. As shown in Figures 3A–E, SPOCK2 mRNA expression level was significantly correlated with patient’s race (Caucasian vs. African-american, *p* < 0.01) and tumor grade (Grade 2 vs. Grade 3, *p* < 0.05), and has no relation with patient’s age, individual cancer stage, and TP53 mutation status (*p* > 0.05). The univariate analysis with logistic regression showed that upregulated SPOCK2 mRNA expression is positively associated with tumor residual (OR = 1.746 for RD vs. NRD, *p* = 0.045) (Table 1). Furthermore, we found that protein expression level of SPOCK2 was positively associated with tumor grade (Normal vs. Grade 2, *p* < 0.001; Normal vs. Grade 3, *p* < 0.01), patient’s race (Caucasian vs. Asian, *p* < 0.01), and individual cancer stage (Stage 1 vs. Stage 4, *p* < 0.01; Stage 3 vs. Stage 4, *p* < 0.001) (Figures 3F–H). These results revealed that overexpressed SPOCK2 was susceptible to a more advanced disease and was more common in the Caucasian patients, indicating that SPOCK2 has potentials to be a prognostic indicator for HGSOC patients.

**FIGURE 3:** SPOCK2 expression level in subgroups of patients with HGSOC. Boxplots of SPOCK2 mRNA expression based on patient’s age **(A)**, patient’s race **(B)**, tumor grade **(C)**, cancer stage **(D)**, and TP53 mutation status **(E)**. Boxplots of SPOCK2 protein expression based on tumor grade **(F)**, patient’s race **(G)**, and cancer stage **(H)**. (Significant codes of *p*-value: *, *p* < 0.05; ***, *p* < 0.001).

**TABLE 1:** SPOCK2 expression associated with clinicopathological characteristics.

Characteristics	Total (N)	Odds Ratio (OR)	*P*-value
Age (>60 vs. <=60)	379	1.200 (0.801-1.801)	0.378
Race (Asian and Black or African American vs. White)	365	0.850 (0.426-1.680)	0.640
FIGO stage (Stage III&Stage IV vs. Stage I&Stage II)	376	0.989 (0.428-2.283)	0.979
Histologic grade (G3&G4 vs. G1&G2)	369	1.183 (0.637-2.216)	0.595
Tumor status (With tumor vs. Tumor free)	337	1.126 (0.668-1.903)	0.655
Tumor residual (RD vs. NRD)	335	1.746 (1.018-3.034)	**0.045**
Lymphatic invasion (Yes vs. No)	149	0.938 (0.470-1.868)	0.856
Venous invasion (Yes vs. No)	105	0.587 (0.263-1.290)	0.188
Primary therapy outcome (PR&CR vs. PD&SD)	308	1.323 (0.717-2.473)	0.373

Bold value means significance.

### High SPOCK2 expression is associated with poor prognosis

Kaplan-Meier curves were used to explore the relationships between SPOCK2 mRNA expression and OS in HGSOC patients. As shown in Figure 4A, the result of Kaplan-Meier analysis showed that HGSOC patients with high level of SPOCK2 mRNA expression in the TCGA-OV data set had a worse OS than those with a low expression (HR = 1.45, CI: 1.12–1.88, *p* = 0.005). Next, we performed subgroup survival analyses of OS based on clinical characteristics, which exhibited that prognosis of patients with high-level SPOCK2 expression was significantly poor in the White (HR = 1.44, CI: 1.09–1.89, *p* = 0.01), stage III&IV (HR = 1.48, CI: 1.14–1.92, *p* = 0.004), and Grade 3&4 (HR = 1.47, CI: 1.11–1.95, *p* = 0.007) subgroups of OS (Figures 4D–I). Notably, for HGSOC cases with high-level SPOCK2 expression, patients aged over 60 years (HR = 1.66, CI: 1.15–2.41, *p* = 0.007) and under 60 years (HR = 1.47, CI: 1.02–2.12, *p* = 0.039) both have comparatively worse OS than those with low-level expression (Figures 4B,C). To further find clinical factors associated with survival, we first performed univariate logistic regression analysis which found that age (HR = 1.355, CI: 1.046–1.754, *p* = 0.021), primary therapy outcome (HR = 0.301, CI: 0.204–0.444, *p* < 0.001), tumor status (HR = 9.576, CI: 4.476–20.486, *p* < 0.001), tumor residual (HR = 2.313, CI: 1.486–3.599, *p* < 0.001), and SPOCK2 expression level (HR = 1.445, CI: 1.115–1.872, *p* = 0.005) were significantly associated with OS (Figure 5A, Supplementary Table S1). In addition, multivariate Cox regression analysis showed that primary therapy outcome (HR = 0.365, CI: 0.237–0.563, *p* < 0.001) and tumor status (HR = 19.162, CI: 4.689–78.307, *p* < 0.001) were independent prognostic factors of OS for HGSOC; SPOCK2 expression level, however, was not still an independent factor related to OS (HR = 1.297, CI: 0.939–1.791, *p* = 0.114) (Figure 5B, Supplementary Table S1).

**FIGURE 4:** Kaplan-Meier survival curves comparing the high and low expression of SPOCK2 in HGSOC. Survival curve of OS between SPOCK2-high and -low patients **(A)**. Survival curves of OS between SPOCK2-high and -low subgroups among patients with age≤60 **(B)**, age > 60 **(C)**, White **(D)**, Asian and Black or African American **(E)**, stage I&II **(F)**, stage III&IV **(G)**, Grade 1 and 2 **(H)**, Grade 3 and 4 **(I)**.

**FIGURE 5:** Univariate logistic **(A)** and multivariate Cox **(B)** regression analyses showing hazard ratios (HRs) for different clinical variables.

### Constructing the prognostic models for high-grade serous ovarian cancer

To quantitatively verify that SPOCK2 mRNA is an advisable approach predicting the prognosis of HGSOC patients, SPOCK2 and other clinicopathological parameters including age, FIGO stage, histological grade, and primary therapy outcome were used to construct a prediction model for OS. We, therefore, established a nomogram of OS based on multivariate Cox regression analysis to assign points to the abovementioned variables. The points assigned to these variables were accumulated and recorded as the total score. For example, HGSOC patients with high SPOCK2 mRNA expression (25 points), advanced FIGO stages (59 points), and age over 60 years (19 points) received a total score of 103. Then, we draw a vertical line directly down from the total points axis at scale of 103 to the survival probability axis. Therefore, the 1-, 3-, and 5-years survival probabilities were >95%, 68%, and 36%, respectively (Figure 6A). Moreover, we evaluated the performance of the nomogram by using Calibration curves, and the result showed that C-index of the model was 0.638 (CI: 0.616–0.661), which indicated that the prediction efficiency of this model is moderately accurate (Figure 6B). Overall, these results suggested that the nomogram was a better model for predicting survival in HGSOC patients than individual prognostic factors.

**FIGURE 6:** Quantitative methods to predict HGSOC patients’ 1-, 3-, and 5-years survival probability. A nomogram predicting 1-, 3-, and 5-years survival probability **(A)**. Calibration plots of the nomogram for predicting the probability of OS at 1, 3, and 5 years **(B)**.

### Co-expressed genes of SPOCK2 in high-grade serous ovarian cancer

To explore the co-expressed genes of SPOCK2, we used the LinkFinder module. As shown in the Volcano plot (Figure 7B), a total of 6,453 genes were identified to be significantly correlated with SPOCk2 (*p* < 0.05). Following this, we showed top 50 genes that positively and negatively correlated with SPOCk2 in the heat maps, respectively (Figures 7A,D). In addition, the scatter plots were used to present the most closely correlated genes with SPOCK2, including CRB2 (Pearson-Correlation: 0.606, *p =* 8.543E-32), ARHGAP23 (Pearson-Correlation: 0.533, *p =* 1.247E-23), TGM1 (Pearson-Correlation: 0.532, *p =* 1.518E-23), AKAP7 (Pearson-Correlation: −0.377, *p =* 1.191E-11), and MERTK (Pearson-Correlation: −0.361, *p =* 9.034E-11) (Figures 7C,E–H).

**FIGURE 7:** SPOCK2-correlated genes. All significantly correlated genes with SPOCK2 distinguished by Pearson test **(B)**. Top 50 genes positively **(A)** and negatively **(D)** related to SPOCK2 showed by heat maps. Scatter plots presenting the most closely correlated genes of SPOCk2 with CRB2 **(C)**, ARHGAP23 **(E)**, TGM1 **(F)**, AKAP7 **(G)**, and MERTK **(H)**.

### Functional enrichment analysis of SPOCK2

We used the LinkInterpreter module to explore functional enrichment information of SPOCK2 that contribute to tumorigenesis or tumor progression of HGSOC. KEGG pathway analysis showed that SPOCK2-correlated genes were mainly involved in focal adhesion, leukocyte transendothelial migration, and ECM-receptor interaction (Figure 8A). GO_BP (biological process) was mainly associated with cell junction organization, cell-cell adhesion via plasma-membrane adhesion molecules, and extracellular structure organization (Figure 8B). GO_CC (cell component) was mainly related with extracellular matrix, actin cytoskeleton, contractile fiber, and cell-substrate junction (Figure 8C). GO_MF (molecular function) was mainly associated with extracellular matrix structure constituent, extracellular matrix binding, actin binding, cell adhesion mediator activity, cell adhesion molecule binding, and growth factor binding (Figure 8D). Overall, these top KEGG and GO enrichment items suggested that SPOCK2 might play an important role in modulating extracellular matrix.

**FIGURE 8:** Functional enrichment of SPOCK2-correlated genes. Kyoto encyclopedia of genes and genomes (KEGG) **(A)**, biological process (BP) **(B)**, cell component (CC) **(C)**, and molecular function (MF) **(D)** pathway analyses.

### Immune infiltration analysis of SPOCK2

Given the fact that immune infiltration is deeply involved in anti-tumor responses, we investigated the relationships between expression level of SPOCK2 mRNA and abundance of TILs. First, the heat map showed Spearman correlations between 28 kinds of immune cells and SPOCK2 mRNA expression in 30 TCGA cancer types, which was downloaded from TISIDB (Figure 9A). For HGSOC, correlations between 24 TIL types and SPOCK2 were analyzed by using ssGSEA and the Spearman method (Figure 9B). The scatter plots indicated that SPOCK2 mRNA expression positively correlated with infiltration of natural killer (NK) cells (*R* = 0.310, *p* < 0.001), T effector memory (Tem) cells (*R* = 0.220, *p* < 0.001), T central memory (Tcm) cells (*R* = 0.190, *p* < 0.001), and Mast cells (*R* = 0.110, *p* = 0.033); by contrast, SPOCK2 mRNA expression negatively correlated with infiltration of activated dendritic cells (aDC) (*R* = −0.170, *p* = 0.001) and T helper 2 (Th2) cells (*R* = −0.140, *p* = 0.005) (Figures 9C–H). In addition, the Wilcoxon rank sum test was applied to further verify the correlations between SPOCK2 expression and abovementioned TILs. The plots confirmed that patients in SPOCK2-high group had more NK cells (*p* < 0.001), Tem cells (*p* < 0.01), and Tcm cells (*p* < 0.05), and had less aDC (*p* < 0.01) and Th2 cells (*p* < 0.01); however, the plot showed no significant difference of Mast cells infiltrating abundance between SPOCK2-high and -low groups (*p* > 0.05), which is not consistent with the result of scatter plot (Figure 10). These results manifested that SPOCK2 might have double-edged functions in coordinating the induction of TILs.

**FIGURE 9:** Correlations of SPOCK2 expression with immune infiltration level. Relations between SPOCK2 expression and tumor infiltrating lymphocytes (TILs) across human cancers **(A)**. Correlations of SPOCK2 expression with TILs in HGSOC **(B)**. SPOCK2 expression positively correlated with natural killer (NK) cells **(C)**, T effector memory (Tem) cells **(D)**, T central memory (Tcm) cells **(E)**, and Mast cells **(F)**; by contrast, SPOCK2 expression negatively correlated with activated dendritic cells (aDC) **(G)** and T helper 2 (Th2) cells **(H)**.

**FIGURE 10:** Abundance of NK **(A)**, Tem **(B)**, Tcm **(C)**, Mast **(D)**, aDC **(E)**, and Th2 **(F)** cells between SPOCK-low and -high groups.

## Discussion

In this study, we found that both mRNA and protein expression of SPOCK2 were upregulated in ovarian serous cystadenocarcinoma along with a high expression of SPOCK2 mRNA in the most TCGA cancers. Further ROC curve analysis confirmed that SPOCK2 could be a promising diagnostic biomarker to distinguish HGSOC from benign tissues. To investigate factors that influence SPOCK expression, subgroup analyses based on clinical variables were done in all patients enrolled in the UALCAN dataset, suggesting that SPOCK2 expression is correlated with patient’s race, tumor grade, and cancer stage. A critical element of this study is the evaluation of the effect of SPOCK2 on OS by using Kaplan-Meier and univariate logistic regression analyses, in which high SPOCK2 mRNA expression is associated with a shorter OS. Additionally, functional enrichment analysis of SPOCK2-correlated genes revealed that SPOCK2 may play a specific role in regulating functions of extracellular matrix. Exploratory analyses of TILs were conducted to examine the role of SPOCK2 in immune infiltration, showing that there were significant associations between SPOCK2 mRNA expression level and TILs abundance. Overall, this study has led to an improved understanding of SPOCK2 in HGSOC and provided potential therapeutic target.

SPOCK family comprised of SPOCK1, SPOCK2, and SPOCK3, and was originally identified by cDNA cloning, with amino acid homologies (Vannahme et al., 1999; Bradshaw, 2012). SPOCK proteins share a unique N-terminal region, followed by a follistatin-like (FS) domain, calcium-binding (EC) domain, thyroglobulin type-1 (TY) domain, and a C-terminal tail encompassing heparan/chondroitin sulfate glycosaminoglycan attachment sites at two serine residues (Alliel et al., 1993; Bonnet et al., 1996; Krajnc et al., 2020). To connect protein functions to the spatial organization of SPOCK2 protein domains, Krajnc et al. (2020) confirmed that the FS-EC-TY domain triplet formed a structure core and was responsible for executing functions. All three SPOCKs are extracellular proteoglycans highly expressed in brain, ovary, lung, testis, prostate, and kidney, and it is expected that SPOCKs might contribute to extracellular matrix and associate with tumor progression (Alliel et al., 1993; Bonnet et al., 1996; Vannahme et al., 1999). To gain insight into the biological functions of SPOCKs in human cancers, we focused on SPOCK2 as a presentative of the family because of its upregulated expression and prognostic potential in HGSOC patients (Ren et al., 2011). Nordgard et al. first described the correlation of SPOCK2 with human cancer and found that oligonucleotide polymorphism of SPOCK2 gene was associated with deletion of 16q chromosome in breast cancer (Nordgard et al., 2008). Encoded by the SPOCK2 gene, it is a 424-amino acid protein with a C-terminal tail that binds to glycosaminoglycans to form proteoglycans (Vannahme et al., 1999). In addition to being structural components of extracellular matrix, proteoglycans can serve as important biochemical signals that regulate cell proliferation, differentiation and migration, and modulate vascular networks and immune cell infiltration (Gordon-Weeks and Yuzhalin 2020). Thus, it is essential to determine whether abnormal changes of SPOCK2 exist in HGSOC and how its properties influence tumor progression.

By analyzing the expression level of SPOCK2 in HGSOC, we noted that both mRNA and protein level of SPOCK2 in HGSOC were significantly higher than those in normal ovary tissues, which were influenced by clinical features such as patient’s race, tumor grade, and cancer stage. Few studies have been conducted to explore the underlying reasons of why these clinical characteristics could change genetic performance of SPOCK2. Nevertheless, some studies have focused on mechanisms of up- and down-regulated expression of SPOCK2 and concluded that promoter methylation of SPOCK2 gene may be one of reasons for abnormal expression of SPOCK2. Ren et al. (2011) carried out a retrospective study to compare the protein expression level and methylation status of SPOCK2 in malignant ovarian tissues and benign tissues. They found that the frequency of SPOCK2 hypermethylation in malignant ovarian tissues (45%) was significantly higher than 6.7% in the benign tissues; synchronously, the loss rate of SPOCK2 protein in malignant ovarian tissues was 44%, which was significantly higher than 13.3% in the benign tissues, indicating that SPOCK2 hypermethylation might lead to loss expression of protein. Alternatively, Chung et al. (2008) verified that treatment with 5-aza-2′-deoxycytidine, a demethylating agent, could restore expression of SPOCK2, suggesting that DNA methylation is related to transcriptional silencing of SPOCK2 in prostate, colon, and breast cancer. In addition to DNA methylation, future researches could focus on other epigenetic modifications to figure out how SPOCK2 expression in HGSOC is upregulated.

SPOCK2 was highly expressed in HGSOC patients and was related to poorer OS. This study has, therefore, characterized SPOCK2 mRNA expression as a prognostic biomarker for prognosis. On the contrary, Lu et al. (2021) found that overexpressed SPOCK2 was significantly associated with better OS (HR = 0.302, *p* = 0.016) in patients with pancreatic ductal adenocarcinoma. Similarly, an *in vitro* experiment revealed that overexpression of SPOCK2 contribute to inhibit cell proliferation and invasion in endometrium-derived cancer cell lines. The researchers also found that inhibitory functions of SPOCK2 on tumor cell progression were achieved partly through suppressing expression or activation of MT1-MMP and MMP2 (Ren et al., 2020). However, another *in vitro* study confirmed that abundant distribution of SPOCK2 may contribute to glioma invasion by countering the inhibitory action of SPOCK1 and SPOCK3 and supporting MT-MMP-mediated cell migration (Nakada et al., 2003). In summary, these findings suggested that functions of SPOCKs may differ among human cancers. Although SPOCK2 protein was upregulated in HGSOC, high expression of SPOCK2 protein failed to be a prognostic indicator in this study. Considering that SPOCK2 is a potential biomarker for OS, a nomogram was constructed to predict 1-, 3-, and 5-years survival possibility. Our findings indicated that this nomogram model could help to differentiate more advanced HGSOC patients and determine more aggressive therapeutic regimens.

Functional enrichment analyses in this study demonstrated that biological processes of SPOCK2 in HGSOC often require gene network interactions. To further understand biological capabilities of SPOCK2 in HGSOC, correlated genes were used to perform functional enrichment analysis, finding that SPOCK2 may participate in extracellular matrix structure constituent, focal adhesion, cell junction organization, and growth factor binding. According to the results of previous studies, degradation of extracellular matrix surrounding focal adhesion sites played an important role in regulating metastatic process, which required the proteolytic activity of MT1-MMP. Researcher further verified that focal adhesion kinase (FAK), a focal adhesion component, was essential to recruit MT1-MMP molecules (Wang and McNiven 2012). Moreover, Nakada et al. (2003) found that SPOCK2 could abolish inactivation of MT1-MMP and MT3-MMP by other SPOCK family members and permit migration of glioma cells in the presence of SPOCK1 and SPOCK3 proteins. Accordingly, SPOCK2 could promote remodeling of extracellular matrix and, therefore, was considered as an important molecule in cell migration. Overall, SPOCK2 played critical role in tumor development, suggesting that more future researches would be needed to explore properties of SPOCK2 in HGSOC.

During cancer progression, tumor cells can establish an overtly immunosuppressive tumor microenvironment that is composed of infiltrating immune cells, endothelial cells, and fibroblasts, often embedded within extracellular matrix (Anderson et al., 2017). Numerous studies indicated that abundance of tumor infiltrating immune cells is closely correlated with clinical survival (Hao et al., 2020a; Hao et al., 2020b). However, extracellular matrix surrounding the tumor islets can integrate and deliver multiple complex signals to leukocytes that affect their biological functions, thereby indicating that the complex relationships between extracellular matrix and TILs should be addressed (Pickup et al., 2014). Extracellular matrix can exert antineoplastic activity through providing migratory highways on which leukocytes can directly invade into inflammation-inflamed tumor areas in response to chemo-attractant matrix molecules released *via* MMP-mediated degradation (Sorokin, 2010; Pickup et al., 2014). In this regard, SPOCK2 could promote leukocyte migration and activate anti-tumor inflammation because its facilitative role of MT-MMP-mediated proteolysis that releases chemo-attractant fragments. Similarly, this study found that SPOCK2 positively correlated with infiltration of NK cells, Tem cells, Tcm cells, and Mast cells, indicating a pro-immunogenic role of SPOCK2. Besides inducing anti-tumor immunity, extracellular matrix can directly inhibit T cell activity through impairing the process of antigen presentation (Meyaard, 2008; Vesely et al., 2011). Coincidentally, we found that SPOCK2 negatively correlated with infiltration of aDC which is the most capable antigen-presenting cells, suggesting a pro-tumoral role of SPOCK2. According to published studies, immunosuppressive tumor microenvironment is an unavoidable obstacle to explore effective cancer immunotherapies for patients with ovarian cancer. This redundant immunosuppressive network may facilitate tumor progression by either restraining endogenous antitumor immunity or reducing the quantity of immune cells (Odunsi 2017). On the basis of our findings and previous studies, we concluded that effects of abnormal SPOCK2 expression on TILs still remain elusive, appealing to more fundamental researches.

This study provided evidence for upregulated expression of SPOCK2 and found that SPOCK2 had diagnostic and prognostic potential for HGSOC. In addition to explorations of SPOCK2-related pathways that indicated a critical role in remodeling extracellular matrix, immune cell infiltration analyses provided new understandings for associations between SPOCK2 and TILs. Although a lack of *in vivo*/vitro experiments and use of public databases make it difficult to detail the mechanisms of SPOCK2 that contribute HGSOC progression, this article is expected to provide a new direction for predicting prognosis and exploring therapeutic targets. In the future, more fundamental experiments with clinical samples instead of data mining should be well-designed.

## Data Availability

The original contributions presented in the study are included in the article/Supplementary Material, further inquiries can be directed to the corresponding author.
